The article "Prognostic factors for long-term mortality after surgery of left-sided infective endocarditis" was published in 2025. Journal: PLoS One.

# Prognostic factors for long-term mortality after surgery of left-sided infective endocarditis

**DOI:** 10.1371/journal.pone.0321068

**Published:** 2025-03-31

**Authors:** Se Ju Lee, Jung Ho Kim, Yongseop Lee, Sangmin Ahn, Jung Ah Lee, Jinnam Kim, Hyung Jung Oh, Jin Young Ahn, Su Jin Jeong, Jun Yong Choi, Joon-Sup Yeom, Nam Su Ku, Seung Hyun Lee

**Affiliations:** 1 Division of Infectious Diseases, Department of Internal Medicine and AIDS Research Institute, Yonsei University College of Medicine, Seoul, Republic of Korea; 2 Division of Infectious Diseases, Department of Internal Medicine, Inha University College of Medicine, Incheon, Republic of Korea; 3 Department of Internal Medicine, Hanyang University College of Medicine, Seoul, Republic of Korea; 4 Division of Nephrology, Sheikh Khalifa Specialty Hospital, Ras Al Khaimah, United Arab Emirates; 5 Division of Cardiovascular Surgery, Severance Cardiovascular Hospital, Yonsei University College of Medicine, Seoul, Republic of Korea; Children's National Hospital, George Washington University, UNITED STATES OF AMERICA

## Abstract

**Background:**

Infective endocarditis has low prevalence but a high mortality rate. Left-sided infective endocarditis (LSIE) has a higher mortality rate than right-sided infective endocarditis. Surgical treatment is occasionally considered for LSIE; however, few data are available on the long-term prognostic factors for LSIE after surgical treatment. This study investigated the risk factors for long-term mortality in LSIE patients who underwent surgical treatment.

**Methods:**

This retrospective study enrolled adult patients with LSIE who were admitted to Severance Hospital in South Korea and underwent surgical treatment from November 2005 to August 2017. The primary outcome was risk factors for overall all-cause mortality. Multivariable Cox regression analysis was performed to identify risk factors for long-term mortality of patients with LSIE who received surgical treatment.

**Results:**

This study enrolled 239 with LSIE who underwent surgery. The median follow-up period was 75.9 months, and there were 34 deaths (14.2%) during the study period. Multivariable Cox analysis showed that central nervous system complications (hazard ratio [HR]: 3.55, 95% confidence interval [CI]: 1.76–7.17, *P* <  0.001), chronic liver disease (CLD) (HR: 4.33, 95% CI: 1.57–11.91, *P* =  0.005), and age ≥  65 years (HR: 2.65, 95% CI: 1.28–5.51, *P* =  0.009) were risk factors for overall mortality. Kaplan–Meier analysis indicated a significant difference in survival between patients with and without CNS complications (*P* <  0.001, log-rank).

**Conclusion:**

Central nervous system complications, CLD, and older age were associated with long-term mortality in surgically treated patients with LSIE. Preventive strategies for CNS complications would improve the treatment of LSIE.

The article "Prognostic factors for long-term mortality after surgery of left-sided infective endocarditis" was published in 2025. Journal: PLoS One.

## Introduction

Infective endocarditis (IE) has low prevalence; however, its incidence is increasing worldwide as a result of advances in diagnostic techniques including cardiac echocardiography and other noninvasive cardiac imaging modalities, increased blood culture sensitivity, and changes in diagnostic criteria [1–3]. This increase may also be influenced by the rising number of patients at elevated risk of endocarditis, due to the increasing number of invasive procedures and the use of prosthetic valves and indwelling cardiac devices [2,4,5]. Despite advances in treatment, the mortality rate of patients with endocarditis has not improved, remaining at 15–30% [6,7].

Left-sided IE (LSIE) and right-sided IE (RSIE) have different characteristics and rates of invasive disease [8]. LSIE has a higher mortality rate than RSIE [7]. RSIE accounts for only 5–10% of IE, and approximately 90% of patients can be treated medically [7]. Surgical treatment is indicated for patients with IE who have heart failure and uncontrolled infection, and to prevent embolism. Surgical treatment can be considered for LSIE and is associated with an improved prognosis [9–12]. Age, diabetes mellitus, and renal dysfunction are associated with adverse outcomes after surgery for patients with LSIE [13–16]. Nonetheless, few data are available on the long-term prognostic factors for LSIE after surgical treatment. Therefore, this study evaluated the risk factors for long-term mortality among patients who received surgical treatment for LSIE at a tertiary hospital in South Korea.

## Materials and methods

### Study population

This retrospective study enrolled adult patients with IE who were admitted to Severance Hospital, a tertiary hospital in South Korea, from November 2005 to August 2017. IE was defined as definite or possible according to the 2000 modified Duke criteria [17]. Patients who met the following criteria were included in the study: >  17 years of age, diagnosed with IE and admitted to Severance Hospital, aortic or mitral valve involvement, and surgical treatment. Patients with pulmonary or tricuspid valve involvement were excluded. The Institutional Review Board of Yonsei University Health System Clinical Trial Centre approved this study (no. 4-2018-0248). Because the study was retrospective and the data were anonymized, the IRB waived the requirement for informed consent. The data were accessed for research purposes on September 20, 2019, and researchers did not access the information that could identify individual participants during or after data collection.

The article "Prognostic factors for long-term mortality after surgery of left-sided infective endocarditis" was published in 2025. Journal: PLoS One.

### Outcomes and variables

Relevant clinical and laboratory data were collected from electronic medical records. Laboratory tests were investigated based on the date of IE diagnosis. The primary outcome was risk factors for long-term mortality in patients with LSIE who underwent surgical treatment. The mortality data was obtained from the Ministry of the Interior and Safety of South Korea, which collects death-related information for all South Korean citizens, to analyze long-term overall mortality. Mortality data were collected up to September 18, 2019. The Charlson comorbidity index was calculated at admission to classify the patients according to their comorbidities. Sequential Organ Failure Assessment (SOFA) scores were used to assess the severity of organ dysfunction. European System for Cardiac Operative Risk Evaluation (EuroSCORE) II scores were calculated to assess cardiac surgical risk [18]. Systemic embolic complications comprised pulmonary embolism, splenic infarction, coronary embolism, and peripheral limb embolism. Central nervous system (CNS) complications comprised ischemic complication, cerebral hemorrhage, cerebral abscess, and intracranial mycotic aneurysm.

### Statistical analyses

The study population was divided into two groups according to death. Differences in patient characteristics and outcomes between the two groups were assessed using the chi-squared test or Fisher’s exact test for categorical variables and the *t*-test or Wilcoxon rank-sum test for continuous variables. Continuous variables were checked for normal distribution using the Shapiro–Wilk test. Adjusted Cox regression analysis was performed to assess the risk factors for long-term mortality of surgically treated LSIE. Variables with *P* <  0.05 in univariate analyses were entered into the multivariable Cox model. Hazard ratios (HRs) and 95% confidence intervals (CIs) were calculated based on the multivariable model. Survival analysis was performed using the Kaplan–Meier method and log-rank test to estimate long-term outcomes according to risk factors identified by the multivariable Cox model. Significance was determined at a level of P <  0.05. All statistical analyses were performed using R v4.2.2 (R Core Team, Vienna, Austria).

## Results

During the study period, 400 adult patients with IE were identified. Among these, 259 patients underwent surgery, and 20 were excluded because of pulmonary or tricuspid valve involvement. Finally, 239 patients were analyzed in this study (median age, 53.0 years; interquartile range [IQR], 40.0–63.0; males, 69.9%). The median follow-up period was 75.9 (IQR, 47.2–108.6) months.

The article "Prognostic factors for long-term mortality after surgery of left-sided infective endocarditis" was published in 2025. Journal: PLoS One.

### Patient characteristics

As of September 2019, 34 patients had died. The survival group was significantly younger (51.0 years: IQR, 39.0–61.0 vs. 61.0 years: IQR, 53.0–72.0, *P* =  0.001) and had lower Charlson comorbidity index (1.0; IQR, 0.0–3.0 *versus* 3.0; IQR, 1.0–5.0, *P* =  0.001), SOFA (1.0: IQR, 1.0–2.0 vs. 2.0: IQR, 1.0–4.0, *P* =  0.014), and EuroSCORE II (1.9: IQR, 1.5–2.8 vs. 2.4: IQR, 2.1–5.1, *P* =  0.001) scores than the mortality group (Table 1). The rate of isolated mitral valve involvement was significantly lower in the mortality group (52.7% vs. 29.4, *P* =  0.02). The frequencies of chronic kidney disease (CKD) (3.9% vs. 17.6%, *P* =  0.007), chronic liver disease (CLD) (3.4% vs. 14.7%, *P* =  0.017), and CNS complications (26.8% vs. 58.8%, *P* <  0.001) were significantly higher in mortality group. The time from diagnosis to surgery did not differ significantly between the two groups (8.0 days: IQR, 4.0–15.0 vs. 11.5 days: IQR 5.0–24.0, *P* =  0.226). There was no significant difference in the rate of pathogen isolation between the two groups (*P* =  0.147).

**Table 1:** Characteristics of surgically treated LSIE patients.

	Survival (n = 205)	Death (n = 34)	*p*-value
Age, years	51.0 (39.0–61.0)	61.0 (53.0–72.0)	**0.001**
Age ≥ 65 years	40 (19.5%)	15 (44.1%)	**0.003**
Male sex	141 (68.8%)	26 (76.5%)	0.482
Community-acquired IE	187 (91.2%)	29 (85.3%)	0.441
Valve status			0.382
Native	183 (89.3%)	28 (82.4%)	
Prosthetic	22 (10.7%)	6 (17.6%)	
Involved valve			
Isolated aortic	57 (27.8%)	14 (41.2%)	0.168
Isolated mitral	108 (52.7%)	10 (29.4%)	**0.020**
Bivalvular involvement	40 (19.5%)	10 (29.4%)	0.277
Comorbidities			
Previous IE	8 (3.9%)	2 (5.9%)	0.638
Predisposing valve condition	79 (38.5%)	17 (50.0%)	0.283
Patients with previous valve surgery or prosthesis	28 (13.7%)	8 (23.5%)	0.218
Patients with cardiac devices	1 (0.5%)	1 (2.9%)	0.265
Diabetes mellitus	30 (14.6%)	8 (23.5%)	0.289
Chronic heart failure	8 (3.9%)	3 (8.8%)	0.194
Chronic kidney disease	8 (3.9%)	6 (17.6%)	**0.007**
Chronic liver disease	7 (3.4%)	5 (14.7%)	**0.017**
Solid cancer	14 (6.8%)	2 (5.9%)	>0.99
Hematologic malignancy	1 (0.5%)	0	>0.99
Immunosuppressive therapy	5 (2.4%)	0	>0.99
Charlson comorbidity index	1.0 (0.0–3.0)	3.0 (1.0–5.0)	**0.001**
Recent antibiotics use	20 (9.8%)	4 (11.8%)	0.757
Modified Duke criteria			
Definite	172 (83.9%)	29 (85.3%)	>0.99
Possible	33 (16.1%)	5 (14.7%)	>0.99
Pathogen			0.147
MSSA	9 (4.4%)	3 (8.8%)	
MRSA	3 (1.5%)	2 (5.9%)	
Streptococcus	94 (45.9%)	9 (26.5%)	
Enterococcus	14 (6.8%)	4 (11.8%)	
Other	24 (11.7%)	6 (17.6%)	
Unknown	61 (29.8%)	10 (29.4%)	
C-Reactive Protein, mg/L	47.3 (10.5–81.6)	61.3 (20.2–138.0)	0.123
SOFA score	1.0 (1.0–2.0)	2.0 (1.0–4.0)	**0.014**
Complication			
CNS complication	55 (26.8%)	20 (58.8%)	**<.001**
Ischemic complication	54 (98.2%)	19 (95.0%)	
New conduction abnormality	16 (7.8%)	4 (11.8%)	0.661
Days to surgery after diagnosis	8.0 (4.0–15.0)	11.5 (5.0–24.0)	0.226
Emergency or urgent vs non-urgent surgery			0.764
Emergency or urgent surgery	63 (30.7%)	9 (26.5%)	
Non-urgent surgery	142 (69.3%)	25 (73.5%)	
EuroSCORE II	1.9 (1.5–2.8)	2.4 (2.1–5.1)	**0.001**
Antibiotics days	31.0 (26.0–41.0)	36.5 (22.0–45.0)	0.987
Antibiotics days after surgery	21.0 (14.0–28.0)	16.5 (7.0–30.0)	0.091
Reoperation	7 (3.4%)	1 (2.9%)	>0.99

* Continuous variables were described as median (interquartile range), and discrete variables were described as numbers (percentages).

The article "Prognostic factors for long-term mortality after surgery of left-sided infective endocarditis" was published in 2025. Journal: PLoS One.

LSIE, left-sided infective endocarditis; MSSA, methicillin-susceptible Staphylococcus aureus; MRSA, methicillin-resistant Staphylococcus aureus; SOFA, Sequential Organ Failure Assessment; CNS, central nervous system.

### Factors associated with long-term mortality

Univariate Cox analysis showed that patients with CNS complications, higher SOFA scores, CLD, CKD, older age, and isolated mitral involvement had significantly higher risk of long-term mortality (Table 2). Multivariable analysis showed that CNS complications (adjusted HR 3.55; 95% CI, 1.76–7.17; *P* <  0.001), older age (adjusted HR 2.65; CI 95%, 1.28–5.51; *P* =  0.009), and CLD (adjusted HR 4.33; 95% CI, 1.57–11.91; *P* =  0.005) were significantly associated with long-term mortality in surgically treated LSIE patients. Kaplan–Meier survival curves for long-term mortality differed significantly according to the presence of CNS complications (Fig 1) (*P* <  0.001, log-rank test).

**Table 2:** Cox regression analysis for long-term mortality.

	Univariate analysis		Multivariable analysis	
	Hazard ratio (95% CI)	*p-*value	Hazard ratio (95% CI)	*p-*value
CNS complication	3.48 (1.76-6.9)	<.001	3.55 (1.76–7.17)	**<.001**
Chronic liver disease	5.01 (1.89-13.2)	0.001	4.33 (1.57–11.91)	**0.005**
Age ≥ 65 year	3.21 (1.62-6.36)	0.001	2.65 (1.28–5.51)	**0.009**
Isolated Mitral valve involvement	0.40 (0.19-0.83)	0.014	0.48 (0.22–1.06)	0.068
SOFA score	1.36 (1.16-1.59)	<.001	1.21 (0.96–1.51)	0.101
Chronic kidney disease	4.65 (1.88-11.49)	0.001	1.33 (0.40–4.41)	0.643

* Continuous variables were described as median (interquartile range), and discrete variables were described as numbers (percentages).

CNS, central nervous system; SOFA, Sequential Organ Failure Assessment; CI, Confidence interval.

**Fig 1:** Kaplan-Meier survival curve for overall mortality according to the CNS complication. CNS, central nervous system.

The article "Prognostic factors for long-term mortality after surgery of left-sided infective endocarditis" was published in 2025. Journal: PLoS One.

## Discussion

CNS complications, older age, and CLD were significantly associated with overall mortality after surgical treatment for LSIE. Neurologic complications are prevalent in IE, and symptomatic CNS complications occur in approximately 35% of patients with IE [19]. The inclusion of asymptomatic CNS complications increased the rate of CNS complications. It has been reported that 82% of patients with IE had cerebral lesions, as assessed by brain magnetic resonance imaging [7,20]. Misfeld *et al*. showed that the long-term prognosis of patients with IE with asymptomatic cerebral embolism was similar to that of patients with symptomatic cerebral embolism [21]. In this study, 31.4% of patients had CNS complications. As in previous reports, ischemia was the most frequent complication.

Prevention of cerebral embolism is an indication for surgery, and neurologic complications are associated with poor outcomes in patients with IE [7,22,23]. The association of neurologic complications with the prognosis of surgically treated LSIE is unclear. Symptomatic neurological complications before surgery in LSIE were found to be significantly associated with a worse prognosis after surgery [24]. A study from Taiwan reported no significant difference in in-hospital mortality rate between surgically treated LSIE patients with and without neurologic complications, possibly because of the small sample size [25]. Carrascal *et al*. reported that patients with LSIE who had preoperative neurological complications and underwent surgery early did not have shorter medium- or long-term survival rates; however, there were trends towards lower medium- and long-term survival rates [26]. The study included only patients with LSIE who underwent early surgery; by contrast, the present study also enrolled non-urgent surgery patients. The risk of CNS complication is highest at the time of diagnosis of IE and decreases after the initiation of antimicrobial therapy [19]. Patients with LSIE on anticoagulants have fewer cerebrovascular accidents (CVA), whereas the effect of anticoagulation on CVA in IE is unclear [27–29]. Consequently, early diagnosis of IE and initiation of antimicrobial therapy are crucial for preventing neurologic complications, which would improve the prognosis after surgery. Physicians’ premature closure of diagnosis reduces the rate of the diagnosis of IE, whereas early obtaining blood culture and recalling the IE diagnosis are helpful in early diagnosis of IE [30,31]. Improving physicians’ awareness of IE and indication of blood culture is important for early diagnosing and treating IE.

In IE, neurologic complications are more frequent in cases of mitral valve involvement than aortic valve involvement [32]. However, in this study, isolated mitral valve involvement tended to be associated with long-term survival. This finding contradicts previous reports that mitral valve involvement is associated with a worse prognosis [32,33]. In this study, patients with isolated mitral involvement tended to be younger (median ages: 47.0, 55.0, and 54.5 years, respectively) and have lower rates of new-onset heart failure (5.1%, 16.9%, and 20.0%) and paravalvular complications (8.5%, 32.4%, and 40.0%) than those with isolated aortic valve or bivalvular involvement. Acute heart failure and paravalvular complications are associated with a worse prognosis in patients with IE [32,34]. These complications might explain the tendency to associate isolated mitral valve involvement with a high overall mortality rate. However, in a multivariable Cox analysis, isolated mitral valve involvement was not significantly associated with long-term mortality.

The article "Prognostic factors for long-term mortality after surgery of left-sided infective endocarditis" was published in 2025. Journal: PLoS One.

CLD is associated with a poor prognosis in IE [35]. Patients with liver cirrhosis have a poor prognosis because of gut bacterial overgrowth and translocation, immune dysfunction, and decreased filtration by the liver [36,37]. In the absence of cirrhosis, chronic infection with hepatitis B virus or fatty liver disease can cause immune suppression, and the result of the present study that chronic liver disease is associated with long-term mortality in patients with LSIE who underwent surgery is consistent with prior reports [38,39].

Patients with IE are typically young [2]. However, as life expectancy increases and risk factors for IE such as DM, cancer, and degenerated valve disease become more prevalent, the average age of IE patients has increased [2,3]. Older age is associated with adverse outcomes after cardiac surgery; in this study, older age was significantly associated with overall mortality after surgical treatment [13,14]. As a result of concerns about complications after surgery, elderly patients with IE tend to receive medical rather than surgical treatment [6,13]. However, Ragnarsson *et al*. reported that surgical treatment was associated with better long-term survival irrespective of age [9]. Therefore, surgical treatment should be considered for elderly patients with IE.

This study had several limitations. First, because it was retrospective, unidentified confounding variables may have affected the results. Second, the pathogen could not be identified in 29% of patients, and inappropriate antimicrobial treatment may have affected the prognosis. However, because the proportion of patients with unknown pathogens in the survival and mortality groups was similar, a significant effect on the results is unlikely. Third, functional status after CNS complications is associated with the long-term prognosis [40]. Therefore, analysis stratified by functional status would provide insight into the effect of CNS complications on the long-term prognosis of LSIE. There are insufficient studies on the long-term survival of patients with IE, particularly on those who undergo surgery, making this study`s findings both novel and useful.

The article "Prognostic factors for long-term mortality after surgery of left-sided infective endocarditis" was published in 2025. Journal: PLoS One.

## Conclusions

In conclusion, CNS complications, CLD, and older age were associated with long-term mortality in patients with LSIE who underwent surgical treatment. Preventive strategies for CNS complications are needed to improve the treatment of LSIE. Further research on means of preventing CNS complications is warranted.
